# Construction and Analysis of College English Teaching Path under the Multiple Network Teaching Environment and Credit System

**DOI:** 10.1155/2022/9841977

**Published:** 2022-08-30

**Authors:** Bin Chong, Zhongshan Tian

**Affiliations:** College of Foreign Languages, Inner Mongolia University of Technology, Hohhot, Inner Mongolia 010051, China

## Abstract

With the wide spread of the Internet, information technology begins to enter all aspects of people's lives, such as teaching. The trend of economic globalization and export-oriented economic development have put forward urgent requirements for the level and quality of English teaching in colleges and universities. However, the current diversified information technology has brought many opportunities and challenges to college English teaching, and the traditional teaching mode can no longer meet the requirements of the new era. Both teachers and students need to communicate and interact through modern network media. Teaching reform has become an inevitable trend. The important premise of deepening college English teaching reform under the credit system is to grasp the needs of students. This paper analyzes the characteristics of the interactive teaching mode, points out the problems and challenges of the traditional English teaching, reveals the achievements and the problems of the reform under the credit system, and concludes that the English teaching mode, which is a practical and effective teaching mode.

## 1. Introduction

With the rapid development of the Internet, information technology has also been widely used in college English teaching [1]. The trend of economic globalization and export-oriented economic development have put forward urgent requirements for the level and quality of English teaching in colleges and universities. The teaching of the newcurriculum should be based on modern information technology, especiallyInternet information technology, break through the conventional teaching methods in the past classroom, and enhance the autonomy of teachers. Therefore, how to form diversified teaching methods will be the key to the reform of College English Teaching [2].

In English classroom teaching, there is a lack of interaction between teachers and students. The specific performance is that the teacher blindly explains in the classroom, while the students can only passively accept, and the two sides rarely communicate. Even if the teacher occasionally asks some questions, it is often quick to give answers, students lack the opportunity to think and participate, the overall classroom is very boring, and students lack interest. The advancement of teaching reform is naturally even more difficult to mention. The Internet, on the other hand, is highly interactive. The state's basic regulations on the macrodevelopment strategy of higher education have pointed out the direction for the reform of college English teaching [3].

The credit system is an important measure in the reform of higher education teaching in China. As a teaching management system, it has undergone a process of continuous improvement, the reform of college English teaching is the proper meaning of the reform of the credit system, and improving the “comprehensive application ability of English” of college students is still the main direction of college English teaching reform. Then, through years ofcredit system education reform, from credit, class hours, subjects, students'independent learning to teaching mode, curriculum focus, teaching resources andteaching management, our main opinions and ideas on the reform of CollegeEnglish curriculum still need to be clarified [4]. Through in-depth research, it is necessary to grasp the psychology of students' needs [5]. After research, it isnecessary to grasp the psychological needs of students [5]. Therefore, we have carried out a specialresearch activity in a certain university with the theme of “CollegeEnglish Teaching Reform under the credit system”, and on this basis, wehave introduced several main inspirations from the questionnaire survey tofurther reform the College English classroom [6].

At present, the research results of foreign language researchers on blended English teaching mostly focus on the theoretical discussion of the effectiveness of blended learning methods in College English teaching; Or, pay attention to the interaction with learners in the mixed learning model; English teaching model, as well as the use of academic Various modes can realize the integration of online and offline learning from a macro perspective, but do not give a detailed description from a micro perspective [7]. The specific courses of College English majors and their guiding role deserve further study [8].

Wen Qiufang (2013) put forward the “output-driven hypothesis” for formal foreign language classroom teaching: (1) In terms of the teaching process, the output is greater than the input in foreign language learning, as shown in Figure 1. (2) As far as teaching objectives are concerned, cultivating expressive language skills in speaking, writing, and translating is more in line with social needs. Therefore, the expressionskills of spoken, written and translated texts are all explicit evaluationgoals, while the acceptance skills of hearing and reading are implicit goals [9]. According to the specificrequirements of social occupation, college students can choose one or severalmajor abilities in oral, writing and reading as the selection task [10].

## 2. State of the Art

### 2.1. The Theoretical Basis of the Multi-Interactive Teaching Mode

#### 2.1.1. Constructivist Learning Theory

Constructivist learningtheory provides the most intuitive conceptual support for the multipleinteractive teaching mode, while constructivistlearning theory focuses on how to internalize the object learning frameworkinto the subject cognitive framework through personal interaction with theobject learning structure. Constructivists point out that knowledgerefers to the process activities that learners actively deal with knowledge andreconstruct the meaning of knowledge in specific social life scenes on thebasis of their own cognitive experience and experience [11]. The application of constructivist learning theory to college English teaching means that learners are not passively accepting knowledge objects, but actively acquiring knowledge and constructing new meanings [12]. In this process, they musttruly internalize their professional knowledge into their own language abilitythrough their own practice. However, the traditional teaching methods oflanguage courses in Colleges and universities in China have not achieved thisgoal well. Since the previous English Teaching in Chinamainly focused on teaching language theoretical knowledge, teachers generallyuse abstract words and sentences that are far away from the context as analysismaterials, and let learners carry out rational syntactic analysis beforeEnglish-Chinese translation. Therefore, this teaching method limits theirknowledge creation skills and language communication skills, The most importantfactor is to affect their learning enthusiasm and subjective initiative. At the same time, we should focus on collaborative learning so that students can gain more knowledge [13].

#### 2.1.2. Self-Directed Learning Theory

Autonomous learning theoryrefers to the behavior of students as the main body of learning. They can actindependently without being restricted by others or influenced by the outsideworld, and complete their studies by reading, listening, experiment, readingand experiment. In the 1980s, Henri Holecbrought the idea of active education into foreign language teaching [14]. Since the rise of the ideaof autonomous learning, many experts have carried out in-depth research on itin different aspects. Therefore, the autonomous learning strategies in OxfordUniversity mainly include perception strategy, memory strategy, compensationstrategy, metacognitive strategy, emotional strategy and social strategy.Although scholars have different views, scholars generally believe thatautonomous learning must take learners as the core, and learners should buildsystems through different behaviors and complete planning, autonomousmanagement, autonomous adjustment, autonomous detection, autonomous responseand self-evaluation in the whole perceived environment [15], as shown in Figure 2.

### 2.2. The Characteristics of the Multi-Interactive Teaching Mode

The multiple interactiveteaching mode is an organic system composed of the relationship between theeducational environment and the teaching subject, and is an innovative teachingmethod that conforms to the modern educational reform and development trend. There is a big difference between the multi-interactive teaching mode and the traditional teaching mode, as shown in Table 1.

 The rapid development of modern computer technology has provided the necessary conditions for therealization of synchronous and asynchronous communication between teachers and students in schools, and thus computer communication in a real degree can be realized [16]. As shown in Figure 3, an integrated interactive teaching platform can be built through the network. This process involves thecommunication between teachers in the classroom, teachers after class, studentsand schools, including learning media and teaching resources. This continuum includes teacher-student interactions in the classroom, teacher-student interactions outside the classroom, student-student interactions, and student interactions with learning media and learning materials [17].

Various mobile APPs for practicing vocabulary, reading, listening, and speaking can help students increase their interest in English learning and further tap their English learning potential, as shown in Figure 4.

## 3. Methodology

The construction of the university English classroom teaching model requires an effective understanding and analysis of the relationship between the various constituent elements, and if you want to do this work well, you must collect, summarize, and integrate all kinds of data and data. On the basis of big data, the collection, induction, and collation of various data and materials can be completed through the following ways, namely, collecting all data related to teaching and learning in and out of the classroom, as well as data related to practice, in addition, collecting online data related to English teaching, but also collecting data related to teaching systems and multimedia, and integrating these data and information at the same time.

In order to solve the twoissues of “what impact does the multi-dimensional interactive teachingmode have on students' English learning” and “what attitude dostudents have towards this teaching mode”, the project selects twoteaching groups with similar disciplines in one college and one school.  Figure 5 shows the specific contents of the learning and memory information processing model [18]. After collecting various data and integrating and summarizing at the same time, it is necessary to analyze the various factors involved in the construction of the English ecological classroom teaching mode with the help of the analysis function of the big data technology itself so as to ensure that the factors can establish a good relationship with each other. As the experimental class(46 students) and the control class (44 students), after completing the lastassessment at the beginning of the grade, they carried out a one semestermultimedia interactive course practice with the practice group [19]. The teachers of theexperimental class guide the students to make learning plans and record thespecific contents and processes of learning in the form of learning files. Atthe same time, the teacher divided the students into three to four teachinggroups, and each group was responsible for teaching demonstration and dramaperformance. Students must work, consult materials, do PowerPoint and completetask rehearsal before teaching. In the activities of communicating and workingwith the organization personnel, the learners not only improve theircommunication skills, but also enhance their English level. Teacherscommunicate and interact with them continuously through our school's learningsystem, QQ, wechat and other Internet development tools, and guide them to dotheir homework, formulate plans, master goals and time, etc. at the same time,they enable them to achieve independent learning through some mobile phone softwareafter class, and then register their learning progress on the archive [20].

## 4. Result Analysis and Discussion

### 4.1. Data Collection and Analysis

The specific operational content of the collection and induction of various types of teaching materials and information mainly includes the following aspects: (1) In the teaching after class, it is necessary to fully understand the specific situation of the students taught by the teaching teacher and the teaching content, methods and methods, student situation, online English teaching, and student participation; (2) in the learning and practice activities after class, the students' written and oral communication ability, the ability to communicate with others in English, the ability to read and write in independent English, and so on; and (3) in the English teaching system, in multimedia data and online data, it is necessary to understand the university English learning materials, English teaching system, the latest micro-lessons, audio and video, English audio materials, and so on. In general, in the process of data collection and collation, we must ensure the immediacy, accuracy, and comprehensiveness of data collection to the greatest extent, which are the prerequisites for realizing the construction of the university English ecological teaching model. Through a week of classroomhows that the posttest scores of boexperiments, we have conducted the second assessment on the students in theexperimental class and the control group, and passed spss19. hows that the posttest scores of boTable 2 shows the results of the two classes. There was no significant difference in English scores in the initial test (*p*-value greater than 0.05); the standard error deviations of the means are 1.56630 and 1.32057, respectively. However, according to Table 3 the scores of the students in the experimental class and the control class after the test are higher than those before the test. However, from the independent sample *t*-test analysis of the total scores of the two classes after the test, although there is no statistically significant difference, the *p*-value has decreased, which also shows that the difference between them is increasing. Perhaps because the experiment lasted only one academic year and the duration was too short, it could not show too obvious difference in performance. However, we can still see that the performance of the experimental class is much better than that of the control class.

### 4.2. Questionnaire and Interview Results

Thisstudy also carried out a simple social survey on the students of the educationexperimental class to understand the impact of multiple interaction modes onstudents' learning, and selected some students for interviews to understand thestudents' understanding and attitude towards these modes. The results are asfollows.

First,the impact of multiple interaction models on students' autonomous learningability: about 67% of students feel that they can establish academic goals andlearning plans under the guidance of teachers; Seventy three percent of thestudents thought that they could better use the online teaching platform andmobile devices such as smart phones or laptops to complete independent learningafter class; And 68% of the students thought they could better cooperate withthe members of the organization.

Second,their understanding and views on the multi language interactive teaching model:84% of the students believe that this teaching model can enhance students'English reading comprehension and can be maintained for a long time; And about12% of the students believe that this teaching mode adds extra time to theiractivities. Academic burden may not be suitable for students; Four percent ofthe students think it doesn't matter which teaching method they adopt.

### 4.3. Credit System Questionnaire Collection and Data Analysis

The experimental subjects were 109 non-English majors: 1 experimental class with 55 students and 1 control class with 54 students. - The two classes adopted thefull credit system. Although they came from different disciplines, the averagescores of the first test were 69.06 and 68.12 respectively. The independentsample t-test results show that there is no significant difference in theaverage English scores between the two classes (*t* = 6.49, *p* > 0.05). The mean scores of the final test were 77.76 and 72.92, respectively, with a significant difference (*p* < 0.05).

### 4.4. Credit System Research Results

#### 4.4.1. Description of Some Questionnaire Results

1. Recognition of the teaching model of “micro-class + flipped classroom”: 72.73% like it; 27.27% dislike it. Some students who choose not to like it think that they have increased the amount of learning and have too high requirements for autonomy.
2. Regardingthe improvement of self-ability under this teaching mode, most people thinkthat the most important thing is the ability to search for materials (73.33%),that is, information literacy; Secondly, the ability to use Englishcomprehensively (70.91%), the ability to produce ppts (66.67%), the ability tocooperate (60%), the ability to make public speeches (56.36%) and so on, inorder to meet the research expectations, and at the same time, the ability touse information, the ability to use English comprehensively and the ability tooutput resources independently.

#### 4.4.2. Description of the Interview Results

In the interview, thestudents of the experimental group gave positive comments, saying that theEnglish class was flexible, interesting, simple and effective, and fullymobilized the students' interest and initiative in learning.The students in the control group thought that the class was boring, monotonous, and the class was too large.

#### 4.4.3. Classroom Observation Description

Thecomprehensive application level of the control group is better than that of thecontrol group, which mainly reflects the use scale, frequency and quality inthe review process. After the end of the semester, the teachers of the classcollected and counted their usual classroom activities and information recordedin the online review system. The results showed that in the control group,everyone participated in the classroom teaching activities 16 times, and basicallyevery lesson content had the opportunity to be published once in the group orschool; In online reading, each person reads more than 30 times, repeats morethan 32 times, and extracts more than 20 times. In the same academic year, eachperson in the control group participated in classroom teaching activities 1.5times, with a single content type, mainly to solve the problems of textvocabulary, after-school exercises and reading in school textbooks.

### 4.5. Suggestion

#### 4.5.1. The Positive Role of Multiple Interactive Teaching Models

Todayis an era of rapid development of information and constant updating of scienceand technology. Therefore, machine learning knowledge can neither meet theneeds of learners for knowledge nor adapt to the fierce international competitionin the future. Autonomous Learning and lifelong learning are both related tothe sustainable development of learners and the ability of continuousself-improvement. The multi-dimensional interactive teaching mode enablesstudents to understand various teaching methods, especially metacognitivestrategies and social methods, through deep-seated and multi-dimensionalcommunication in class and after class, online and offline, so as to improvestudents' active learning ability.

#### 4.5.2. Challenges Brought by Multiple Interactive Teaching Models

Ifthe multi teacher interaction mode is not properly used, it will produce amultiplier effect of 0.5. Therefore, teacher cooperation is required to bebetter applied.

Firstof all, there are higher requirements for teachers. We need to screen morenetwork resources, optimize the curriculum, and set up interactive topics andexchange projects according to the characteristics and acceptance of differentgrades. In addition, even in extra-curricular life, teachers must useface-to-face teaching or online Q & A to constantly monitor and helpchildren's review and academic progress.

Otherwise, it is easy for students to be in a state of laissez-faire.

Second, there is more needfor students' self-learning consciousness. Some students have a weak foundationand may have many difficulties in autonomous learning activities. Therefore,their extracurricular interactive learning requires them to further enhancetheir self-monitoring ability to understand various learning strategies andreading methods and cooperate with each other.

Third,there are higher requirements for the software and hardware construction of thecampus. Teachers' interactive teaching and students' autonomous learning alsoneed to have relatively complete educational software and hardware equipment oncampus, including campus autonomous learning system, autonomous learningclassroom and other educational facilities. In particular, the popularity ofmobile phones requires a complete Internet signal on campus.

The fourth is to further improvethe diversified assessment system. In the multi interactive teaching method,the result evaluation method that only focuses on teaching results and neglectsthe learning process is no longer suitable, so the evaluation means must bemore perfect. The evaluation subject and evaluation means should also bediversified to reflect the development process of teaching results andcommunication process, so as to realize active learning for learners.

#### 4.5.3. Implications of the Credit System

Basedon the comprehensive consideration of the psychological characteristics ofCollege English Teaching under the credit system, the following suggestions areput forward to further promote the reform of College English Teaching:

1.Adjust the subject setting and further optimize the teaching materials. The newschool score system reform will be implemented in an all-round way to promotethe further adjustment of school teaching and the further optimization ofteaching materials. The school-hour humanities elective course is divided intoseven compulsory courses: “translation and writing, cross-culturalcommunication, English newspaper selection, high-end English audio-visual, English professional film and television appreciation, Chinese local cultureEnglish professional learning guide and high-end oral English”. Theseseven compulsory courses are also called “comprehensive applicationcompulsory courses for College English Majors”. They are built according tothe characteristics of local culture and economic development, Strive tocultivate the overall application skills of international communication throughEnglish Majors in the period of rapid social and economic development. In 2009, the comprehensive application course for English Majors in Colleges anduniversities was listed as the “national excellent teachingmaterial”. The compulsory courses of general higher education under thecredit system in Colleges and universities take “College English Majors” (1 to 4) as the classroomteaching object, which conforms to the “basic provisions” in theprofessional standards of the National Academic Affairs Office. If thispositioning was feasible two years ago, the current practice proves that it hasnot reached the best state. As only 15% of the students can participate in the “College English major application elective course”, the rest canonly study the “College English major” (1-4). Obviously, thesesituations can not meet the characteristics of the information age and the needsof learners. “College English application course” must be offered tolearners in an all-round way. In order to improve the teaching effect, collegesand universities may issue corresponding regulations. In addition, strongcharacteristic application projects can be set up to meet the needs of learnersin various disciplines and stages.
Innovating teaching mode and strengtheningclassroom teaching for a long time, English Teaching in Chinese colleges anduniversities has always implemented the teaching mode of teaching based onteaching. Although we advocate interactive teaching mode, due to the size of the class. to the real place. With the rapid development of computer, a new teachingmethod is proposed for computer-aided education. When the credit system isimplemented, on the premise of small class hours and large school scale,teachers must adopt modern teaching mode and actively explore and innovatetraditional teaching mode. Multimedia means, vivid, vivid and intuitive. Thenetwork can not only present rich, novel, real-time and colorful educationalresources, but also contact teachers and schools, students and students,Chinese and foreigners. Thislively, interesting and lively teaching mode and teaching method plays a vitalrole in cultivating students' interest in learning, enlightening learners'minds, broadening learners' horizons and enhancing teaching effects.
Toimprove the quality of teachers and pay attention to the education art creditsystem, the marginal problems of English teaching reform in schools are notonly for schools, but also for all teachers. Only by strictly requiring oneselfto master and change one step ahead of the students, and becoming a pioneer andguide in the forefront of English teaching reform, can we carry out moreeffective teaching reform in the interaction between teachers and students.First, improve the concept of teaching reform. According to the provisions ofthe Ministry of education on the teaching requirements of English courses inordinary colleges and universities and the needs of the reform and developmentplan of higher education for the socialist legal construction in China, and the requirements of the national medium and long-term educationreform and development plan, and focus on the goal of quality education andtraining high-level English talents. Establish correct College English teaching concepts and promote thedevelopment of College English teaching reform. Second, we should improveteachers' various qualities and levels. The quality and level of teachers is aprocess determined by many factors. If students have excellent ideological andmoral cultivation, they must pay attention to carrying forward the main melodyof Chinese language and culture education, and have the ability and consciousnessto identify excellent civilization and backward culture. Basic knowledge,technical ability and psychological quality related to the characteristics ofEnglish teaching; Strengthen the ability of information retrieval, processingand evaluation, and good scientific research and innovation ability. Thequality and ability of English teachers in a school directly affect whether theteaching reform can be carried out smoothly. Third, attach importance to theart of education. Such as the art of cultivating students' interest in learningand active learning, the art of cultivating students' creative spirit andinnovative ability, the art of improving teachers' classroom effectiveness, andthe art of improving students' practical and cross-cultural communicationability..
It is a complex and richproject to reform the teaching management mode and promote the mechanismteaching. The reform of College English teaching has provided many new problemsto the teaching management, which requires scientific and reasonable contentsetting and mechanism research in many important subjects of teachingmanagement. First, it has formed a dynamic mechanism for the survival of thefittest. The competitive mechanism of students' learning should be included inthe dynamic control of the curriculum, instead of requiring them to take theexamination for life after entering the school. Instead of judging heroes bytheir achievements or setbacks, we should pay more attention to learners'continuous learning. Improve innovation ability. The second is to build alearner oriented teaching organization system that is conducive to cultivatingstudents' learning interests, such as various English academic interest groupsystems, network teacher communication systems, and student participation incommunity practice systems. The third is to build a teacher training managementsystem, that is, a management system for improving professional ability throughtraining, a scientific research training management system, a trainingmanagement system for improving quality through the use of computer networkinformation technology, and a management system for studying abroad. The fourthis to build a teacher performance evaluation system. Through research andapplication of statistical technology, it can comprehensively and objectivelytest learners' English effect, assess teachers' teaching methods, and assessthe management of relevant units. It must be noted that the system innovationand mechanism innovation of English teaching management in Colleges anduniversities are a whole, covering all important aspects of colleges anduniversities, including educational ideas, teaching processes, teaching models.A detailed explanation will be given.

## 5. Conclusion

With thevigorous development of the Internet, modern information technology has alsobeen more and more widely used in English Teaching in Chinese colleges anduniversities. New teaching methods should be based on modern informationtechnology, especially Internet information technology, and improve teachers'initiative by breaking through conventional classroom methods, but deepen the reform of college English teachingcredit system under the important premise is to grasp the needs of students.Thecomparative analysis of the characteristics of the interactive teaching modeand the traditional teaching mode presents the problems of the traditionalEnglish teaching and the new result. This study has great significance to theconstruction of the network teaching environment and the English teaching modeunder the credit system.

## Figures and Tables

**Figure 1:** Schematic diagram of the graded teaching system of college English.

**Figure 2:** Learning is integrated in three universal processes: information, methods, and cognition.

**Figure 3:** Multiway interaction platform based on the network.

**Figure 4:** Deep learning implementation process.

**Figure 5:** Gagne's information processing model of learning and memory.

**Table 1:** Comparison of traditional teaching mode and multi-interactive teaching mode.

	Traditional teaching mode	Multiple interactive teaching mode
Teacher role	Imparter of knowledge	Knowledge inspirer
Student role	Passive recipient of knowledge	Interactive event participants
Teaching method	Lecture-based	Teachers design interactive topics, learn
Class interaction	There is a small amount of teacher-student interaction in the classroom	Students participate in the interaction
	Traditional teaching mode	Multiple interactive teaching mode
Interactive way	Classroom lectures	Interact at any time through the internet before, during, and after class
Interactive medium	Less used	Network media, such as QQ, WeChat, online learning platforms, etc.
Feedback	Mainly assignments or quizzes	Conduct communication and feedback at any time
Evaluation method	Summative evaluation is the main method, ignoring the personality differences of students	Give priority to formative evaluation, and focus on diversified evaluation
Advantage	Systematic explanation of knowledge, easy for teachers to control the classroom	Flexible and diverse teaching forms, students are highly motivated and involved
Limitation	Low student engagement	Teacher workload increases

**Table 2:** Early statistics for test scores.

Class	*N*	Mean	Std	Standard error of the mean	*t*	Sig (both sides)
Experimental class	46	35.22	10.623	1.56630	0.41	0.968
Control class	44	35.13	8.759	1.32057		

**Table 3:** Statistics of posttest scores.

Class	*N*	Mean	Std	Standard error of the mean	*t*	Sig (both sides)
Experimental class	46	42.99	11.0540	1.62983	1.033	0.304
Control class	44	40.56	11.2578	1.69718		

## Data Availability

The labeled dataset used to support the findings of this study is available from the corresponding author upon request.
